The article "Comparison between the Radiographic and Clinical Rates of Success for TheraCal and MTA in Primary Tooth Pulpotomy within a 12-Month Follow-Up: A Split-Mouth Clinical Trial" was published in 2023. Journal: Biomed Res Int.

# Comparison between the Radiographic and Clinical Rates of Success for TheraCal and MTA in Primary Tooth Pulpotomy within a 12-Month Follow-Up: A Split-Mouth Clinical Trial

**DOI:** 10.1155/2023/8735145

**Published:** 2023-04-19

**Authors:** Sedigheh Hassanpour, Naser Asl Aminabadi, Mahdi Rahbar, Leila Erfanparast

**Affiliations:** ^1^Department of Pediatric Dentistry, School of Dentistry, Bandar Abbas University of Medical Sciences, Bandar Abbas, Iran; ^2^Department of Pediatric Dentistry, Faculty of Dentistry, Tabriz University of Medical Sciences, Tabriz, Iran; ^3^Department of Restorative Dentistry, School of Dentistry, Ardabil University of Medical Sciences, Ardabil, Iran

## Abstract

**Background:**

The present study was conducted for contrasting the efficacy of TheraCal and MTA for primary molar pulpotomy.

**Methods:**

During the current split-mouth randomized clinical trial, 90 bilateral primary molars from 45 healthy 5- to 8-year-old children were pulpotomized using TheraCal in one bilateral tooth and MTA in the other, randomly. Glass ionomer (GI) was used to cover these materials. Then, the treated teeth were restored with stainless steel crowns (SSC) and followed up clinically and radiographically at months 6 and 12 after treatment for any pulpotomy failure indications. Finally, data were analyzed by chi-square test considering *p* value < 0.05 as statistically significant.

**Results:**

Among 82 teeth available at the final follow-up session, the total success rates were 98.1% and 99.3% for TheraCal and MTA, respectively, showing no significant difference between the two groups (*p* > 0.05).

**Conclusion:**

TheraCal can be used as an alternative material for pulpotomy of primary teeth instead of MTA.

## 1. Introduction

Pulpotomy is a clinical procedure widely applied for treating exposed pulps due to caries. After pulpectomy treatment, the radicular pulp should be kept vital, uninfected, and enclosed in the dentin chamber using a dressing material [1].

In the recent decades, MTA has been the gold standard material for pulp capping of primary molars after pulpotomy [2]. MTA has also antimicrobial properties and a dentinogenic effect on the pulp tissue by inducing the release of cytokines from the bone cells that stimulate hard tissue formation [3–5]. In addition, MTA preserves the integrity of pulp tissue with no cytotoxic effect [6]. However, the clinical application of MTA has got limited by some properties such as its long-time setting [6, 7], difficult handling [8], being washed out [9], discoloration, and its high price [5, 10].

Recently, a newer resin-based material has been introduced for endodontic treatments: TheraCal. This light-cured Portland cement-based resin consists of tricalcium silicate particles in a hydrophilic monomer that imitates the hydroxyapatite structure. Also, releasing calcium ions by TheraCal stimulates secondary dentin formation, as well as cell growth and proliferation [11]. Compared to MTA and other traditional materials based on calcium hydroxides (Ca(OH)_2_), TheraCal is less soluble, and its handling is easier, can be dispensed from a syringe, and releases higher calcium ions [12]. Handling TheraCal requires no mixing, clicking, or triturating. Then, it can be precisely placed and immediately set in the pulp chamber [11, 13].

Overall, the findings on using TheraCal compared to other standard biomaterials including MTA have been promising, and it is a potential bioinductive agent that can be easily applied especially in pediatric patients. Accordingly, this study is aimed at evaluating and contrasting the success rates of TheraCal and MTA in terms of clinical and radiographic outcomes of pulpotomies in primary molars. This study was designed as a split-mouth randomized controlled clinical trial with two follow-up sessions after 6 and 12 months.

## 2. Materials and Methods

This study was approved by the Ethics Committee of Tabriz University of Medical Sciences (approval no. IRCT20100125003168N7, 12 March 2019) and is compatible with the Helsinki Declaration of Human Rights. The study was carried out in Pediatric Dentistry Department, Dental Faculty, Tabriz University of Medical Sciences, starting on 23 March 2019 and continuing until 21 March 2020.

### 2.1. Sampling

The study group consisted of 45 patients aged 5-8 years old referring to the Department of Pediatric Dentistry for routine dental treatment. The inclusion criteria were (a) general physical and mental health; (b) healthy gingiva and periodontium; (c) no confounding medical history; (d) no pathologic symptoms including spontaneous pain, tooth mobility, redness, vestibulum swelling, root resorption, and draining sinus tracts; (e) no sensitivity to palpation in the vestibule; (f) no radiolucency observed in furcal and periapical regions; and (g) no pathology observed in the permanent tooth follicles.

Written informed consents were obtained and recorded from all parents/legal guardians for participating in this project and to be available during the 12-month follow-up. They were all informed about the study procedure, possible risks, and discomforts, as well as the expecting benefits.

### 2.2. Sample Size

To calculate the appropriate sample size, 20 pulpotomized primary molars were treated with TheraCal and MTA and then were followed up for three months. In terms of pain as the primary subsequence, a 12% outcome difference was observed between the two materials. Therefore, considering *α* = 0.05, power = 80%, and 25% outcome difference between pulpotomized teeth using TheraCal and MTA, it was concluded that at least 39 teeth in each group were required for this study. However, it was increased to 45 to endorse the power of the study and compensate for any possible inconsistency in the follow-up program.

### 2.3. Clinical Methods

After a comprehensive dental examination, the clinical procedures were carried out in two consecutive sessions. In the initial appointment, children got familiar with the dental environment, instruments, and procedures through the standardized “tell-show-do” method. Thereafter, the children received prophylaxis followed by professional topical fluoride therapy. The next session started with a brief initial communication to establish rapport with the child (using simple statements and questions). Then, a chief postgraduate student provided all dental treatments to all included subjects under the supervision of an experienced pediatric dentist. Treatment included prophylaxis, local anesthesia (2% lidocaine with 1/80,000 epinephrine), TheraCal and MTA pulpotomy (according to the guidelines of the American Academy of Pediatric Dentistry), and SSC placement, respectively.

Since the materials used in the study needed different manipulation techniques, the operator could not be blinded to the treatment. However, all other contributors were kept blinded to the groups and procedures. Anesthesia in all groups was performed using rubber dam isolation. The pulp chamber and vital pulp exposure were obtained after the removal of caries using a #330 high-speed bur with a water spray. Subsequently, the coronal pulp tissue was removed down to the canal perforations using a sterile slow-speed round bur (#6 or #8). Then, irrigation of the pulp chamber was performed using a light water flow followed by evacuation. A sterile cotton pellet soaked in sterile saline was then placed against the stumps of the pulp at the openings of the root canals for a few minutes [14, 15]. After hemostasis, the materials were applied based on the study group as specified below. The bleeding was usually controlled by 5 minutes of pressure with moistened cotton pallet in normal saline. In the cases where the bleeding did not stop, the tooth was excluded from the study and subjected to more extensive treatment. In other subjects with normal blood clotting, sterile saline was used to rinse the pulp chamber to make sure there is no blood clot in the pulp chamber. After hemostasis establishment, the teeth were randomly treated with either TheraCal-LC® (BISCO Inc., Schaumburg, IL, USA) or white MTA (ProRoot; Dentsply, Tulsa, OK, USA). Randomization was performed with RandList software (version 1.2; DatInf GmbH, Tubingen, Germany). The symmetric tooth treatment with alternative experimental material was carried out in another session through the same preparation procedure. The whole procedure was accomplished in one session. Immediately after treatment, periapical radiographs were obtained from each treated tooth.

### 2.4. MTA Group

When hemostasis was established, MTA as a white powder (ProRoot; Dentsply, Tulsa, OK, USA) was prepared as was instructed by the manufacturers and then placed in the pulp chamber using a carrier (G. Hartzell & Son, Concord, CA, USA, #ISS52, 1.8 mm). After, it was gently squeezed with a moist cotton pellet for better adaptation to the pulp chamber. Then, it was covered with a thickness of 2 mm layer of low viscous cement type of GI (Fuji II, GC, Japan) [16]. All teeth were restored with SSC (3M, USA) [17].

### 2.5. TheraCal Group

In this group, TheraCal was placed over the pulp stump after hemostasis in one-millimeter thickness layers and underwent light curing for 20 seconds (Dentamerica, UK) [1]. Thereafter, low-viscosity GI cement was used to fill the remaining space of the pulp chamber, and the tooth restoration was performed by SSC (3M, USA) [17].

### 2.6. Follow-Up Study

Six and twelve months post treatment, patients were recalled for comprehensive radiographic and clinical examinations. Two experienced pediatric dentists were recruited for conducting each follow-up appointment who were blinded to the materials and calibrated with the study in an independent meeting before the follow-up sessions [18]. In every follow-up session, the radiographic and clinical data were evaluated for interexaminer reliability using the kappa agreement coefficient [19]. Presenting either of sinus tract, swelling, periapical lesion, spontaneous pain or long-lasting pain, tenderness to palpation and percussion, internal/external root resorption, or interradicular radiolucency was accounted as the treatment failure. However, these symptoms were ruled out: gingival problem, food impaction, and other similar sources of pain that mimicked irreversible pulpitis. Tenderness to percussion and internal root resorption were considered radiographic and clinical criteria for evaluating the interexaminer reliability using the kappa agreement coefficient [1, 14].

### 2.7. Statistical Analysis

For comparing the qualitative data, chi-square or Fisher's exact tests were used and the Pearson correlation test was applied to compare means. All data analyses were conducted using SPSS 20 software (IBM, Chicago, IL, USA). The *p* value < 0.05 was considered statistically significant.

## 3. Results

In total, 82 primary molars (40 mandibular molars and 42 maxillary molars) received pulpotomy in forty-one 5- to 8-year-old children (mean = 5.5 ± 1.12, 24 females and 21 males). Four patients were excluded due to missed follow-ups or missing data (Figure 1). There was no significant difference in the age and gender of children between the two study groups at the baseline and 12-month follow-up (Table 1). In Figure 1, the flow of participants from the baseline to the final follow-up session (after 12 months) and the reasons for dropouts are also illustrated.

Excellent agreement between the examiners was shown at the baseline (0.93) and follow-ups after 6 months (0.90) and 12 months (0.90) using overall Cohen's kappa coefficient. Also, no statistical difference was shown among their evaluations (*p* > 0.05).

The radiographic and clinical success rates at 6-month follow-up were shown to be 100% in the MTA group, whereas after the 12-month follow-up, the radiographic and clinical success rates were 98.8 ± 7.7% and 100%, respectively.

The radiographic and clinical success rates at 6-month follow-up in the TheraCal group were 98.9 ± 7.4% and 97.8 ± 14.9%, respectively. Also, widening of PDL, furcal radiolucency, pain, tenderness, abscess, and pathologic mobility were recorded in one (2.2%) case. In the same group, after a 12-month follow-up session, internal resorption, loss of integrity lamina dura, widening of PDL, furcal radiolucency, and tenderness were, respectively, detected in 1 (2.4%), 1 (2.4%), 2 (4.9%), 3 (7.3%), and 1 (2.4%) subjects. Additionally, the radiographic and clinical success rates showed to be 97.2 ± 11.6% and 99.4 ± 3.8%, respectively. Overall, the success rates of pulpotomy with TheraCal were 98.4% after 6 months and 98.1% after 12 months (Table 2).

Comparison of pulpotomy clinical success rate between the MTA and TheraCal groups using the Pearson correlation test revealed no significant differences over both 6-month (*p* = 0.320) and 12-month (*p* = 0.320) follow-up assessments. Also, comparing the pulpotomy radiographic success rates between the two study groups revealed no significant differences in either 6-month (*p* = 0.320) or 12-month (*p* = 0.462) follow-up sessions (Tables 3 and 4).

## 4. Discussion

To the extent of the authors' knowledge, few data are published on the effectiveness of TheraCal in pulpotomy of the primary molar. On the other hand, MTA is considered an ideal material for this purpose having excellent biocompatibility properties. However, its high cost, difficult handling, long setting time, and probability of discoloration have limited its usage expansion [8]. Accordingly, the present study is aimed at comparing TheraCal and MTA for primary molar pulpotomy in a split-mouth randomized controlled clinical trial model. The present findings demonstrated an excellent success rate with TheraCal similar to those reported in the literature with MTA for pulpotomy in a primary molar. The overall success rates were 99.3% and 98.1% in the MTA and TheraCal groups after the 12-month follow-up, respectively.

In the current study, MTA was applied as the control because of the numerous properties that have made it the gold standard material for pulpotomy in primary teeth. Its features include biocompatibility, bioinductivity, physical strength, antimicrobial effects, and proper sealing [2, 16, 20, 21].

According to the findings from the used evaluative methods in our study, the MTA-treated primary molars showed a 100% clinical success rate at both 6-month and 12-month follow-up sessions. To the present findings, some other studies have mentioned similar clinical success rates for the MTA material [22, 23]. MTA's superiority over TheraCal in most clinical outcomes is probably because of its high sealing ability and biocompatibility that lead to hard tissue bridge formation and strong barrier creation against any future microbial permeation into the canals that preserves the remained pulp [24, 25]. On the other hand, the high clinical success rates of TheraCal in our study (99.4%) may be attributed to the cement's bacteriostatic properties which could be because of its high alkalinity.

In both MTA and TheraCal groups, radiographic failures were more common than clinical ones. However, MTA and TheraCal showed no periapical radiolucency. This can be explained by their appropriate coronal seal and high resistance against penetrating bacteria into the periapical areas. Parallelly, GI capped with SSC was used to reduce the microleakage along with the entire restoration interface [21].

Similar to some other studies, no external or internal resorption was observed in the MTA-treated teeth [22, 26]. However, in one TheraCal-treated tooth, internal resorption was observed after 12 months and considered a failure of pulpotomy treatment (Figure 2). The precise reason underlying the internal resorption is not known; however, previous investigations suggest the association of eugenol in ZOE with a risk for subsequent internal resorption [27]. Nevertheless, this cannot explain the internal resorption in the present study because ZOE paste was not used as a base on the pulpal tissue. Another reason suggested for the internal resorption has been overstimulation of the primary pulp by the highly alkaline Ca(OH)_2_ which could lead to the formation of odontoclasts by causing metaplasia within the pulp tissue [11].

The setting mechanism and calcium releasing properties of TheraCal are modified due to the presence of resin matrix in its formulation, for example, lower solubility and higher calcium release compared to the self-setting calcium hydroxide and ProRoot MTA [12]. Also, it has better mechanical properties due to further setting after its initial curing because of water penetration to the hydrophilic resin matrix. TheraCal was a very qualified agent and presented close rates to MTA. The frequency of hard tissue bridge formation in TheraCal was comparable with that of pure Portland cement which is higher in frequency and thickness than glass ionomer and resin-based calcium hydroxide. Interestingly, in our study, calcified bridge formation was observed in radiographies in some of the cases in both groups after 12 months (Figure 3). The concept of dentin bridge formation under pulpotomy medicaments has also remained a debated topic among the researchers who suggest it to be either a healing response or the pulp reaction to irritation [28, 29]. Therefore, dentin bridging cannot be considered a reliable response for the determination of success or failure [30].

The most important concern about biomaterials used in pulpotomy is their biocompatibility and cytotoxicity since the material contacts directly to the pulp. Free uncured resin monomers in resin-modified materials such as TheraCal may have a cytotoxic effect [31]. A reduced polymerization degree may cause elevated uncured resin monomers, which eventually may lower the cement's biocompatibility. In a study by Bakhtiar et al. [32] with a cavity depth of 2 millimeters, TheraCal showed poorer pulpotomy outcomes compared to MTA. To ensure complete curing and prevent the effects of free monomers, we reduced the thickness of the TheraCal to one millimeter. Similar to the study of Lee et al. which used 1 millimeter of cavity depth [31], satisfying pulpotomy outcomes were achieved in our study.

Overall, our findings demonstrated remarkable results of TheraCal in pulpotomy of primary teeth at the 12-month follow-up. Therefore, TheraCal can be considered as an alternative material in the pulpotomy of primary teeth.

Exposure location is an important determining factor; occlusal exposures are more successful than proximal ones. A five-minute guideline is provided by an expert, but there is evidence that failure to control bleeding may lead to reduced success in DPCs and reinforces the need to use direct clinical observation in diagnosis and decision-making. Absence of symptoms and preservation of pulp vitality after at least one year indicates a successful VPT. Another factor that affects the success of direct pulp cap is the ability to control pulpal bleeding after exposure and before pulpal bleeding. If the tooth is asymptomatic and well filled, even if the decay remains, the tooth's chances of survival are excellent [33, 34].

It is important to note the limitations of this study since they can determine the future direction of the present study. Firstly, it was the potential release of free monomers from TheraCal that its effect on reducing the biocompatibility was not well-known. Second, we did not observe the histological quality of dentin bridges under TheraCal. Meanwhile, with the precise histological examination of the treated teeth, a more understanding of the effect of TheraCal in pulpotomy milk teeth can be obtained. Finally, a larger sample size with long-term follow-ups until the exfoliation of treated teeth is suggested to assess the histologic results more accurately in different groups.

## 5. Conclusions

The current study confirmed TheraCal as a promising material for pulp capping in pulpotomy of primary teeth. The successful radiographic and clinical outcomes of TheraCal were repeated here in a 12-month follow-up in agreement with several other studies.

## Figures and Tables

**Figure 1:** Flow chart of participants from baseline to 12-month follow-up.

**Figure 2:** Internal root resorption in the tooth treated with TheraCal after 6 months.

**Figure 3:** Dentin bridge formation in teeth treated with TheraCal (a) and MTA (b) after 12 months.

**Table 1:** Characteristics of the assessed patients and teeth during the follow-ups.

		Follow-up 1		Follow-up 2	
Age		5.5 ± 1.12		5.8 ± 0.7	
Gender	Male	24	53.3%	23	56.1%
	Female	21	46.7%	18	43.9%
Jaw type	Mandible	44	48.9%	40	48.8%
	Maxilla	46	51.1%	42	51.2%
Molar NO	First molar	42	46.7%	38	46.3%
	Second molar	48	53.3%	44	53.7%

**Table 2:** Comparing the findings of 6- and 12-month follow-up sessions between the MTA and TheraCal groups.

Evaluation criteria	After 6 months		After 12 months		Overall
	MTA	TheraCal	MTA	TheraCal	
External resorption	0	0	0	0	0
Internal resorption	0	0	0	2.4	2.4
Loss of integrity of lamina dura	0	2.2	2.4	2.4	7
Widening of PDL	0	2.2	2.4	4.9	9.5
Furcal radiolucency	0	2.2	2.4	7.3	11.9
Periapical radiolucency	0	0	0	0	0
Pain	0	2.2	0	0	2.2
Tenderness to percussion	0	2.2	0	2.4	4.6
Abscess	0	2.2	0	0	2.2
Mobility	0	2.2	0	0	2.2

**Table 3:** Comparing the radiographic success rates of pulpotomy between the MTA and TheraCal groups.

	MTA group		TheraCal group		*p* value
	Mean	SD	Mean	SD	
6-month follow-up	100	0	98.9	7.4	0.320
12-month follow-up	98.8	7.7	97.2	11.6	0.462

**Table 4:** Comparing the clinical success rates of pulpotomy between the MTA and TheraCal groups.

		MTA group		TheraCal group		*p* value
		Mean	SD	Mean	SD	
6-month follow-up	100	0		97.8	14.9	0.320
12-month follow-up	100	0		99.4	3.8	0.320

## Data Availability

The data used to support the findings of this study are included within the article.

## References

[1] Wassel M. O., Amin D. H., Badran A. S. (2017). Clinical, Radiographic, and histological evaluation of TheraCal pulpotomy in human primary teeth. *Egyptian Dental Journal*.

[2] Bossù M., Iaculli F., Di Giorgio G., Salucci A., Polimeni A., Di Carlo S. (2020). Different pulp dressing materials for the pulpotomy of primary teeth: a systematic review of the literature. *Journal of Clinical Medicine*.

[3] TRP F. O. R. D., Torabinejad M., Abedi H. R., Bakland L. K., Kariyawasam S. P. (1996). Using mineral trioxide aggregate as a pulp-capping material. *The Journal of the American Dental Association*.

[4] Oskoee S. S., Bahari M., Daneshpooy M., Ajami A.-A., Rahbar M. (2018). Effect of different intraorifice barriers and bleaching agents on the fracture resistance of endodontically treated anterior teeth. *Journal of Endodontics*.

[5] Parirokh M., Torabinejad M. (2010). Mineral trioxide aggregate: a comprehensive literature review--part I: chemical, physical, and antibacterial properties. *Journal of Endodontics*.

[6] Chng H. K., Islam I., Yap A. U. J., Tong Y. W., Koh E. T. (2005). Properties of a new root-end filling material. *Journal of Endodontics*.

[7] Sluyk S., Moon P., Hartwell G. (1998). Evaluation of setting properties and retention characteristics of mineral trioxide aggregate when used as a furcation perforation repair material. *Journal of Endodontics*.

[8] Johnson B. R. (1999). Considerations in the selection of a root-end filling material. *Oral Surgery, Oral Medicine, Oral Pathology, Oral Radiology, and Endodontology*.

[9] Formosa L., Mallia B., Camilleri J. (2013). A quantitative method for determining the antiwashout characteristics of cement-based dental materials including mineral trioxide aggregate. *International endodontic journal*.

[10] Samiei M., Janani M., Asl-Aminabadi N. (2017). Effect of the TiO2 nanoparticles on the selected physical properties of mineral trioxide aggregate. *Journal of clinical and experimental dentistry*.

[11] Nowak A., Christensen J. R., Mabry T. R., Townsend J. A., Wells M. H. (2018). *Pediatric Dentistry-E-Book: Infancy through Adolescence*.

[12] Gandolfi M., Siboni F., Prati C. (2012). Chemical–physical properties of TheraCal, a novel light-curable MTA-like material for pulp capping. *International endodontic journal*.

[13] Gandolfi M. G., Taddei P., Siboni F., Modena E., Ciapetti G., Prati C. (2011). Development of the foremost light-curable calcium-silicate MTA cement as root- end in oral surgery. Chemical-physical properties, bioactivity and biological behavior. *Chemical–physical properties, bioactivity and biological behavior. dental materials*.

[14] Jamali Z., Alavi V., Najafpour E., Aminabadi N. A., Shirazi S. (2018). Randomized controlled trial of pulpotomy in primary molars using MTA and formocresol compared to 3Mixtatin: a novel biomaterial. *The Journal of clinical pediatric dentistry*.

[15] Tyas M. J. (1998). Pulp protection under restorations - do you need a liner?. *Australian Endodontic Journal*.

[16] Camilleri J. (2014). Hydration characteristics of biodentine and Theracal used as pulp capping materials. *Dental Materials*.

[17] Komabayashi T., Zhu Q., Eberhart R., Imai Y. (2016). Current status of direct pulp-capping materials for permanent teeth. *Dental materials journal*.

[18] Erdem A. P., Guven Y., Balli B. (2011). Success rates of mineral trioxide aggregate, ferric sulfate, and formocresol pulpotomies: a 24-month study. *Pediatric dentistry*.

[19] Cox C., Sübay R., Ostro E., Suzuki S., Suzuki S. (1996). Tunnel defects in dentin bridges: their formation following direct pulp capping. *Operative dentistry*.

[20] Havale R., Anegundi R. T., Indushekar K., Sudha P. (2013). Clinical and radiographic evaluation of pulpotomies in primary molars with formocresol, glutaraldehyde and ferric sulphate. *Oral Health and Dental Management*.

[21] Shih W.-Y. (2016). Microleakage in different primary tooth restorations. *Journal of the Chinese Medical Association*.

[22] Goyal P., Pandit I., Gugnani N., Gupta M., Goel R., Gambhir R. S. (2016). Clinical and radiographic comparison of various medicaments used for pulpotomy in primary molars: a randomized clinical trial. *European journal of dentistry*.

[23] Holan G., Eidelman E., Fuks A. B. (2005). Long-term evaluation of pulpotomy in primary molars using mineral trioxide aggregate or formocresol. *Pediatric dentistry*.

[24] Alqaderi H., Lee C.-T., Borzangy S., Pagonis T. C. (2016). Coronal pulpotomy for cariously exposed permanent posterior teeth with closed apices: a systematic review and meta-analysis. *Journal of dentistry*.

[25] Eskandarinezhad M., Shahveghar-Asl N., Sharghi R. (2017). Sealing efficacy of mineral trioxide aggregate with and without nanosilver for root end filling: an in vitro bacterial leakage study. *Journal of clinical and experimental dentistry*.

[26] Sari Ş., Sönmez D. (2006). Internal resorption treated with mineral trioxide aggregate in a primary molar tooth: 18-month follow-up. *Journal of Endodontics*.

[27] Moretti A., Sakai V., Oliveira T. (2008). The effectiveness of mineral trioxide aggregate, calcium hydroxide and formocresol for pulpotomies in primary teeth. *International endodontic journal.*.

[28] González Rodríguez W. D., Corona Carpio M. H., Martínez Ramos M. R., García Milanés M., Núñez Antúnez L. (2007). Pulpotomies of dead pulps in temporal molars using 10% propolis tinction. *Revista Cubana de Estomatología*.

[29] Silva F. B., Almeida J. M., Sousa S. M. G. (2004). Natural medicaments in endodontics: a comparative study of the anti-inflammatory action. *Brazilian oral research*.

[30] Kusum B., Rakesh K., Richa K. (2015). Clinical and radiographical evaluation of mineral trioxide aggregate, biodentine and propolis as pulpotomy medicaments in primary teeth. *Restorative dentistry & endodontics*.

[31] Lee H., Shin Y., Kim S.-O., Lee H.-S., Choi H.-J., Song J. S. (2015). Comparative study of pulpal responses to pulpotomy with ProRoot MTA, RetroMTA, and TheraCal in dogs’ teeth. *Journal of Endodontics*.

[32] Bakhtiar H., Nekoofar M. H., Aminishakib P. (2017). Human pulp responses to partial pulpotomy treatment with TheraCal as compared with biodentine and ProRoot MTA: a clinical trial. *Journal of Endodontics*.

[33] Edwards D., Stone S., Bailey O., Tomson P. (2021). Preserving pulp vitality: part two - vital pulp therapies. *British Dental Journal*.

[34] Hilton T. J. (2009). Keys to clinical success with pulp capping: a review of the literature. *Operative dentistry*.

